RETRACTED

# Gradual Rarefaction of Hematopoietic Precursors and Atrophy in a Depleted microRNA 29a, b and c Environment

**DOI:** 10.1371/journal.pone.0131981

**Published:** 2015-07-06

**Authors:** Lauren Kauffman, Veronica Balatti, Luciano Cascione, Paolo Fadda, Frederick Racke, Ramasamy Santhanam, Stefan Costinean

**Affiliations:** 1 Department of Pathology, Ohio State Wexner Medical Center, Columbus, United States of America; 2 Comprehensive Cancer Center, The Ohio State University, Columbus, United States of America; 3 Institute of Oncology Research, Bellinzona, Switzerland; Emory University, UNITED STATES

## Abstract

**Background:**

The self-renewing ability of HSCs is fundamental for the maintenance of a pool of bone marrow precursors throughout the life of an individual. The genetic mechanisms underlying such a complex process are still poorly understood.

**Results and Significance:**

Here, we show that constitutive in vivo deletion of miR29ab1 leads to reduced number of HSCs and that miR29ab1 deficient bone marrow cannot repopulate the bone marrow of irradiated mice. An Affymetrix analysis of the miR29ab1 knockout mice identifies key proteins that could be responsible for this phenotype, as DNMT3a and b. Moreover, our findings reveal that whereas miR29b2c knockout mice do not exhibit any spontaneous abnormality, the double knock out – miR29ab1b2c – has marked generalized atrophy, raising the possibility that the two bi-cistrons might cooperate in order to maintain the stem cell number in general, not only limited to the bone marrow.

## Introduction

Hematopoiesis is based on self-renewing hematopoietic stem cells (HSC) and a stepwise process where lineage restricted progenitors generate mature blood cells [1]. Moreover, leukemias are thought to originate from genetically altered stem cells (leukemia stem cells, LSC) [2]. It seems that genes involved in the HSCs maintenance are also relevant for the initiation and progression of leukemias.

The mechanisms underlying HSCs self-renewal are not completely elucidated. Recently, a new class of noncoding genes was identified, called microRNAs [3]. Recent research has shown that microRNA 29a is highly expressed in HSC and AML (acute myeloid leukemia) [4] whereas miR29 is deleted in AML cell lines [5].

Here, we show that constitutive deletion of miR29ab1 leads to gradual rarefaction of HSCs, whereas miR29b2c knockout mice are entirely normal. Colony forming assays at different age points showed consistent decrease of the HSCs in the miR29ab1 deficient mice compared to the wild type littermates. Also, miR29 deficient bone marrow transplants failed to repopulate the bone marrow of irradiated wild type mice. Affymetrix analysis identified upregulated mRNAs like DNMT3a and b in the miR29 knockouts vs wild type littermate controls. MiR29 double knockouts exhibit markedly generalized atrophy.

RETRACTED

This indicates a more general role of the miR29 gene clusters in maintaining the size of viscera through an adequate amount of cellularity.

## Materials and Methods

### Generation of 29ab1, 29 b2c and double knockouts

All procedures were performed in accordance with the Ohio State University Institutional Animal Care and Use Committee-approved protocols. Homozygous floxed miR-29ab1 mice (C57BL6 strain) were generated as follows: for the targeting construct, two homologous recombination arms were amplified by PCR on 129 SvJ/X1 genomic DNA: a 5′ arm of 4171 bp and a 3′ arm of 3857 bp. The genomic fragment to be deleted of 600 bp, containing the miR-29a and miR-29b1, was amplified the same way and cloned in between two loxP sites in a pFlox vector. The recombination arms together with the floxed genes were all cloned into Gateway vectors (Invitrogen) and then assembled together into a destination vector that represented the targeting vector. 129SvJ/X1 ES cells were electroporated with the targeting vector, and clones were screened by Southern blot. DNA was digested with SacI and labeled with a 3′ probe. One positive clone was identified out of 336 screened. The mutant ES cell clone was injected into C57BL/6 blastocysts, and agouti pups were screened by PCR to verify the generation of heterozygous floxed miR-29ab1 mice. Homozygous floxed miR-29ab1 mice were bred to EIIacre mice acquired from Jackson lab to induce ubiquitous deletion of the cluster [6]. The portion of the targeting vector containing neoR is present in the knockout mice. Mir29b2c knockout was obtained in a similar fashion: the 5’ arm was 5007bp whereas the 3’ arm was 4117 bp. The deleted gene fragment was 901 bp. ScaI was used as an enzyme for Southern Blots to differentiate between wild type and heterozygous clones. Three mutated clones were identified out of 336 screened. Homozygous mice were also bred to EIIacre mice [6]. The double knockout was obtained from breeding the two individual knockouts.

### Ethics statement

The Ohio State University Institutional Animal Care and Use Committee (IACUC) specifically approved this study.

### Northern blot

Spleen and liver were dissociated between two frosted slides, and the lysate was washed in PBS, depleted of red cells by hypotonic lysis with ammonium chloride (NH_4_Cl), centrifuged, and resuspended in PBS. Total RNA was extracted with TRIzol (Life Technologies, Invitrogen), loaded and denatured on SDS-PAGE, and blotted on a Hybond N+ membrane (Amersham Pharmacia). The membrane was hybridized with a gamma-^32^P radioactive probe representing the antisense sequence of mature mmu-miR-29a, incubated overnight, washed, and exposed to a PhosphorImager screen (Molecular Dynamics). The image was processed by using a Typhoon image processing system (Amersham Biosciences).

RETRACTED

### RT-PCR for miR29a, b and c

Mature miR29a, b and c (Applied Biosystem) expression was analyzed by Taqman MiR assay and normalized on RNU44 (Applied Biosystem Assay ID: 002750, cat# 4427975) according to the manufacturer’s protocol. 10 nanograms of total RNA from all samples was reverse transcribed for target miR29a, b and c and for the RNU44 housekeeping reference. Samples were analyzed in triplicate and the expression of miR29a, b and c was measured by using the Ct (threshold-cycle) method. The amount of target, normalized to an endogenous reference is given by: 2-ΔCt (Comparative Ct method, Applied Biosystem).

### Histology

Spleens and bone marrow were fixed in formalin, paraffin embedded and cut at 4 microns. Slides were stained H&E. Bone marrow aspirates were Giemsa stained (modified Romanovsky stain)

### Flow cytometry

Single-cell suspension of bone marrow cells was depleted of mature red blood cells by hypotonic lysis (0.165 M NH_4_Cl) and stained with the following conjugated antibodies: anti-B220, CD3, CD117, CD19, IgM, Lys6g and CD11b (all antibodies were from BD Pharmingen). Flow cytometry was carried out on a BD FACSCalibur, and data were analyzed using the BD FACS Convert 1.0 for Mac software.

### Colony forming assay experiments

Bone marrows from miR29ab1 wild type and ko mice were harvested at different ages (2, 6 and 10 months old) and were plated 1X104 cells per plate in Methocult (M3234) suplemented with IMDM plus cytokines [mSCF (10ng/ml) 50ng/ml working conc. mIL-3 (2ug/ml) 10ng/ml mIL-6 (20ng/ml) 10ng/ml h EPO (20,000u/ml)] and 3U/ml L-GLUPen/Strep. Cells were plated in triplicate for each mouse and the colonies were scored after 10days.

### Cytogenetics

Femur bone marrow was flushed with RPMI medium 1640/20% FBS and collected into 5 ml of RPMI medium 1640/20% FBS with heparin 1%. Cells were grown and assessed for chromosomal deletions, translocations, inversions, and number of metaphases.

### Affymetrix

GeneChip Mouse genome 430 2.0 arrays (Affymetrix), containing probe sets for >45,000 characterized genes and expressed sequence tags, were used. Sample labeling and processing, GeneChip hybridization, and scanning were performed according to Affymetrix protocols. Briefly, double-stranded cDNA was synthesized from total RNA with the SuperScript Choice System (Invitrogen), with a T7 RNA polymerase promoter site added to its 3′ end (Genset, La Jolla, CA). Biotinylated cRNAs were generated from cDNAs *in vitro* and amplified by using the BioArray T7 RNA polymerase labeling kit (Enzo Diagnostics). After purification of cRNAs by the RNeasy mini kit (Qiagen, Hilden, Germany), 20 μg of cRNA was fragmented at 94°C for 35 min. Approximately 12.5 μg of fragmented cRNA was used in a 250-μl hybridization mixture containing herring-sperm DNA (0.1 mg/ml; Promega), plus bacterial and phage cRNA controls (1.5 pM BioB, 5 pM BioC, 25 pM BioD, and 100 pM Cre) to serve as internal controls for hybridization efficiency. Aliquots (200 μl) of the mixture were hybridized to arrays for 18 h at 45°C in a GeneChip Hybridization Oven 640 (Affymetrix). Each array was washed and stained with streptavidin—phycoerythrin (Invitrogen) and amplified with biotinylated anti-streptavidin antibody (Vector Laboratories) on the GeneChip Fluidics Station 450 (Affymetrix). Arrays were scanned with the GeneArray G7 scanner (Affymetrix) to obtain image and signal intensities.

RETRACTED

All Affymetrix profile results were uploaded on GEO, at http://www.ncbi.nlm.nih.gov/geo/info/datasets.html.

### In vivo bone marrow transplantations

Five 8- to 15-week recipient mice were irradiated with 1.1 Gy administered in 2 fractions to minimize toxicity. The recipient mice were represented by wild type littermate controls of the miR29ab1 knockouts. T cell—depleted BM cells (5 × 10^6^) from 5 miR29ab1 homozygous knockout and 5 wild type littermate donors were administered via tail vein injection after the radiation. The mice were sacrificed 50 days later using CO_2_ euthanasia chambers (as per the OSU IACUC approved protocol). Bone marrow histological sections and aspirates from the transplanted mice were examined. Specifically, the bone marrow aspirates were used for the evaluation of the bone marrow progenitors and the findings were correlated with the histology and cellularity of the bone marrows.

### Euthanasia method

All mice were sacrificed using CO_2_ euthanasia chambers, as per the OSU IACUC approved protocol.

## Results and Discussion

We generated two distinct miR29ab1 and miR29b2c loxP conditional ko mice without deletion. These were afterwards crossed with EIIA cre mice, which led to the deletion of the two 29 microRNAs clusters during the first couple of weeks of embryogenesis [6]. The heterozygous were then crossed again and pups were checked for complete absence of expression of the genes (S1A and S1B File). Northern Blots and RT-PCRs performed to check for the absence of miR expression in the homozygous for both miR29ab1 and b2c found total absence of miR29a and b in the 29ab1 knockout and lack of miR29c in the miR29b2c knockouts confirming that miR29b transcription comes mostly from the 29b1 gene (chromosome 7) and not the b2 (chromosome 1) [7, 8] (Fig 1 and S1C, S1D and S1E File). In order to generate the mir29ab1 and b2c double knockout we crossed the two individual knockouts. The pups were once again tested for gene and mature sequence lack of expression. MiR29ab1 knockout mice were normal at birth. Over a 2-year span, miR29ab1 homozygous mice were generated at a rate of 10% and had a lifespan decreased to approximately one year (n = 125) versus 2–2 1/2 years for their wild type littermates (n = 392) (Fig 2). These mice exhibited a decrease of spleen size and weight compared to their littermate wild types (S1F File). Histological examination of the spleens and bone marrows showed a decrease of the white pulp, especially granulocytic lineage (Fig 3). The histological data led us to think that miR29ab1 might play a role in the self-renewal and maintenance of HSCs. To test this hypothesis, we designed an in vitro colony forming assay experiment. We harvested the bone marrows of mice at 2, 6 and 10 months of age and plated the HSCs. We then counted the colonies (colony forming units—CFU) formed and noticed that CFUs for all types of precursors (erythroid, granulocytes, macrophages and megakaryocytes) were numerically less represented in the knockouts compared to the wild types (by a ratio of 0.2–0.5 knockouts vs wild types–Fig 4–p = 0.04, n = 4;Fig 5–p = 0.01, n = 8 and Fig 6–p = 0.006, n = 8). Then, we checked the influence age might have on the number of colonies and discovered that the knockout bone marrows were able to partially compensate for the impact of the miR29a and b deficit with time, i.e. the older mice had only a 1–2 fold less CFU-GM compared to the wild types whereas the younger mice had a 5–10 fold difference. Flow cytometry performed on bone marrow hematopoietic cells show a decrease for CD3, CD117, CD19, IgM, Lys6g, B220 but not for CD11b (S1G File, n-10; p = 0.0001). Hence, there seems to be a reduction of precursor and mature forms in the bone marrow for all lineages. We cannot tell whether this is due to miR29a or b as it has already been shown that the mature sequence of mIR29b is transcribed mainly from the 29b1 gene and not b2 [8]. Complete blood counts (CBC) performed on both the knockout and wild type mice showed a slight decrease the white blood cell count (WBC) by a factor of 0.47 and a decrease of total lymphocyte count by a factor of 0.4 (S1H File; n = 3; p = 0.02 for WBC and lymphocyte counts; neutrophil count difference was not statistically relevant). Cytogenetic analysis of several miR29ab1 knockout mice did not reveal any abnormality (S1I File). Affymetrix analysis of mRNA expression in the miR29ab1 knockouts compared to the wild types showed a significant increase in expression of both DNMT3a and 3b (1.06 and 1.04 log fold respectively) together with other WISP1 (a Wnt pathway related mRNA) and Pak6 (Cdc42 related kinase) (S2A File). To ascertain the role of miR29a and b in maintaining the HSCs bone marrow population, we performed a bone marrow transplant experiment where we transplanted the bone marrow of 5 knockouts mice into 2 irradiated mice. We clearly saw a lack of engraftment of the bone marrows of the miR29ab1 ko as compared to the wild types. MiR 29b2c homozygous mice were born at a normal rate of approximately 25%, and had a normal life span (n = 120). They did not exhibit any histological abnormality. Mir29 double knockouts were markedly atrophic with an almost absent white pulp in the spleen (n = 4). Spleens as well as the rest of their internal organs were markedly decreased in size. The homozygous double knockouts were born at a rate of 1% and had a lifespan of approximately one month (S1K File). Histology showed almost absence of the myeloid lineage (S1L File).

RETRACTED

**Fig 1:** Northern Blot for expression of miR29a in the miR29ab1 hetero and homozygous mice (1 –spleen; 2 –liver).

**Fig 2:** Kaplan-Meyer survival chart for 29ab1 ko mice.

**Fig 3:** Histology of the spleen showing reduction of the myeloid lineage in the knockout versus the wild type.

**Fig 4:** Colony forming assay on 2 months old miR29ab1 knockout bone marrows (n = 4; 2 WT and 2 KO; p = 0.04).

**Fig 5:** Colony forming assay on 6 months old miR29ab1 knockout bone marrows (n = 8; 4 ko + 4 wt; p = 0.01).

**Fig 6:** Colony forming assay on 10 months old miR29ab1 knockout bone marrows (n = 8; 4 ko + 4 wt; p = 0.006).

HSCs are, to this date, the only stem cells used in the clinical practice, and, in spite of a plethora of studies, the exact molecular framework of these cells, the mechanism of their renewal and differentiation are still incompletely elucidated.

Our study shows that miR29ab1 deletion results in the diminution of HSCs together with reduction of multipotent and oligo-potent precursors (CFUs) and failure to repopulate irradiated bone marrows in vivo. This is in line with previous studies that demonstrated that overexpression of the miR29a is implicated in the accelerated self-renewal of HSCs and leads to AML [4]. Interestingly, we found that miR29ab1 nullification had the biggest impact on the CFU-GM (granulocytic and macrophagic) populations (0.2 of the wild type levels at 2 months of age) and this difference seemed to decrease with age, becoming 0.4 of the wild type levels at 10 months old. Intriguingly, we also saw a decrease of total lymphocytes in the peripheral blood of the knockouts compared to the wild types (0.68 fold), decrease that was also reported by the authors of the aforementioned paper, even though their mouse model was a miR29a chimera. This was noticed, in addition to the decrease of the WBC count, which was to be expected. Our research does not confirm, at least in a mouse model, previous studies that indicated miR29b down-regulation as implicated in AML [5], even though that might have seemed like an attractive idea, in the light of the 7q deletion related MDS and the fact that miR29ab1 is localized on chromosome 7.

RETRACTED

However, our Affymetrix data seem to confirm many of the miR29a and b targets like DNMTs, especially 3a and 3b, as previously shown [9], interferon activated gene 202B [7], and one member of the Claudin family [10].

Based on the Affymetrix data and previous literature [4, 7, 10] we can surmise that on one hand miR29a deletion might interfere with the HSCs self-renewal through the upregulation of Wnt and CDC42 pathway whereas the absence of miR29b increases the expression of T-bet and interferon gamma in the CD4+ cells sharpening their selectivity for new HSCs which might result in increased auto-deletion of endogenous HSCs (S3A File). One might wonder why we need two clusters (29ab1 and b2c) since 29ab1 seems to fulfill all the functions. As the miR29 double knockout shows, the combined absence of miR29a, b and c leads to extreme atrophy, pointing to the possibility of cooperation between the two clusters with the goal of maintaining the stem cell populations in various organs in the human body.

To the best of our knowledge, our work is the first to show a comprehensive role of miR29ab1 and b2c in multiple in vivo models in the maintenance of HSCs and possibly other stem cell types. While preparing our manuscript, another group published a similar work in the journal Blood, using miR29ab1 knockouts from Belgium [11]. We had no contact with that group and did not know that they were working on the same project. Their work is definitely very thorough; however, we do feel that our paper offers a more complete in vivo picture of the miR29 function. Unlike the aforementioned group, our paper includes the miR29b2c and the double knockout, as well. Moreover, while we show that the miR29b2c knockout does not have the same phenotype as miR29ab1, we also are able to prove that when both miR29 clusters are deleted a marked decrease of organ and body size ensues, accompanied by a far more drastic diminution of the hematopoietic stem cells. Our results seem to be confirmed by recent work that shows miR29 to be involved in organ and body growth [12]. Therefore, we believe that the prior publication by Hu et al only represents a partial depiction of the consequences of miR29 deletion and that our report is a more detailed account to date of the effects of the deletion of not one but both miR29 clusters.

RETRACTED

## Supporting Information

S1 File Mir29ab1 generation strategy (insert: Southern Blot to identify the mutated clones) (Fig A); mir29b2c generation strategy (insert: Southern Blot to identify the mutated clones) (Fig B); Real Time for miR29a in the miR29ab1 knockout mouse (Fig C); Real Time for miR29b in the miR29ab1 knockout mouse (Fig D); Real Time for miR29c in the miR29b2c knockout mouse (Fig E); spleens collected from 4 month old 29 ab1 ko and WT mice (Fig F); flow cytometry on bone marrow of miR29ab1 knockout mice versus wild type for the antibodies indicated in the table (n = 10; 5 wt +5 ko; p = 0.0001) (Table G); complete blood count for miR29ab1 knockout mice versus wild type (Table H);; cytogenetics for miR 29ab1 knockout failed to show any abnormalities (Fig I); Kaplan Meyer survival chart—miR29 double knockouts versus wild types (Fig K); histology of miR29 double knockout spleens show virtually absent myeloid lineage (Fig L).
(DOCX)

S2 File Affymetrix analysis for miR 29ab1 ko mice 8–12 months old(Table A). (XLS)

S3 File Pathway graphic representation showing hypothetical roles of miR29a and miR29b deletion in the decreased of HSCs (Fig A). (PPTX)
